The article "Effect of Simultaneous Multiplane Surgery on Cardiopulmonary Function in Patients with Moderate to Severe Obstructive Sleep Apnea-Hypopnea Syndrome and Its Curative Effect" was retracted in 2023. Reasons: signs of a paper mill; compromised peer review; unreliable results or conclusions.

# Effect of Simultaneous Multiplane Surgery on Cardiopulmonary Function in Patients with Moderate to Severe Obstructive Sleep Apnea-Hypopnea Syndrome and Its Curative Effect

**DOI:** 10.1155/2022/9241635

**Published:** 2022-09-15

**Authors:** Mingjie Gong, Jingwen Shao

**Affiliations:** Department of Otorhinolaryngology-Head and Neck Surgery, Affiliated Hospital of Jiangnan University, China

## Abstract

**Objective:**

To investigate the changes in cardiopulmonary function in patients with obstructive sleep apnea-hypopnea syndrome (OSAHS) by one-stage multiplane surgery.

**Methods:**

70 patients with moderate and severe OSAHS underwent nasal in our hospital from July 2017 to February 2021, palatopharyngeal, and/or tongue operations simultaneously and were followed up for 6 months. The Epworth Sleeping Scale (ESS) scores of patients before and after surgery were compared to observe the surgical efficacy, and the changes in the cardiopulmonary function of patients before and after surgery were detected. The static and dynamic indexes of cardiopulmonary function, respiratory disturbance index (AHI), and blood oxygen saturation (SaO_2_) were compared before and after the operation.

**Results:**

After surgery, all patients' indexes of static lung function were improved compared with that before surgery. After surgery, the percentage of maximal oxygen uptake peak to the predicted value, percentage of oxygen pulse to the predicted value, the ratio of oxygen uptake power, anaerobic threshold, and maximum ventilatory capacity per minute/maximum exercise volume were increased compared with that before surgery, and AHI and SaO_2_ were improved compared with that before surgery.

**Conclusion:**

This study suggests that it is feasible for patients with OSAHS who are unable to tolerate or unwilling to undergo noninvasive assisted ventilation to undergo simultaneous surgery for multiplane stenosis. It can reduce clinical symptoms and improve cardiopulmonary function.

## 1. Introduction

Obstructive sleep apnea-hypopnea syndrome (OSAHS) is the most common form of sleep breathing disorder. It is caused by a variety of reasons. Patients repeatedly suffer from hypoventilation and/or respiratory interruption during sleep, which leads to chronic intermittent hypoxemia, hypercapnia, and sleep structure disorder and further causes a series of the clinical syndrome of pathophysiological changes in the body [1]. The main clinical characteristics of OSAHS are irregular snoring during sleep, a disorder of breathing and sleep rhythm, repeated apnea, and repeated wakefulness. In severe cases, patients suffer from daytime drowsiness, memory loss, and even psychological, intellectual, and behavioral abnormalities [2]. At present, OSAHS is considered a source disease and one of the independent risk factors for coronary artery disease, congestive heart failure, hypertension, and cerebrovascular diseases. OSAHS is characterized by a long course of the disease and prolonged illness. If timely intervention and treatment are not provided, it will eventually cause substantial economic losses or even endanger life. OSAHS can affect people of all ages, especially the elderly. Therefore, early diagnosis of OSAHS, comprehensive assessment of OSAHS conditions and complications, and control of disease burden caused by disease progression from the source are essential.

Current understanding of the disease essence of OSAHS includes the following two aspects: abnormal structure and function of the upper airway and a series of pathophysiological processes of the inflammatory response caused by repeated hypoxia/reoxygenation at night [3]. The nose and pharynx are the main pathological sites of OSAHS, and the causes of the pathological changes include structural changes and functional abnormalities in this part. Meanwhile, the nose and pharynx target organs of various therapeutic methods [4]. The existence of high respiratory resistance in the upper respiratory tract during sleep is the pathophysiological feature of OSAHS. There are two reasons for the formation of upper airway high resistance breathing: upper airway anatomical stenosis and abnormal pharyngeal muscle function.

Studies on cardiac changes in patients with OSAHS have been carried out in an all-around way at home and abroad. The mechanism of cardiac structure and function changes in patients with OSAHS mainly includes the following aspects [5]: (1) The initial factors of OSAHs-related hypertension mainly come from three aspects, namely, substantial intrapleural negative pressure during vigorous breathing, hypoxemia, and repeated awakening. The specific pathophysiological changes that cause hypertension have not been determined. It is believed that the mechanisms that may cause hypertension mainly include activation of the Renin-Angiotensin-Aldosterone System (RAAS) system, hyperexcitation of sympathetic nerves, damage of baroreceptors, increased volume load, obesity, and the role of inflammatory factors [6]. (2) Relationship between OSAHS and cardiac structure and function changes: hypertension can increase cardiac afterload. The left ventricular afterload increased due to the increased left ventricular transmural pressure, which was caused by the dramatic increase of the negative pressure in the pleural cavity caused by forced breathing. The negative pressure increase in the pleural cavity also increases the venous return blood volume, leading to a series of pathophysiological reactions, including right ventricular enlargement, left ventricular septum shift, and left ventricular filling during the diastolic period, and ultimately increasing the left ventricular preload. The combined effect of the increased load before and after OSAHS reduces the stroke volume of patients, and the decrease in the stroke volume of patients is proportional to the negative pleural pressure [7]. The heart and bronchopulmonary tissues are located in the thoracic cavity. Whether the change of pleural pressure will cause the change in cardiac structure remains to be further studied. The pathophysiological basis of cardiac structure and function changes in patients with OSAHS includes wakefulness and nocturnal hypoxia. Therefore, the respiratory function and cardiac changes of patients with OSAHS are the key factors affecting the quality of life of patients and the actual cause of death of patients with OSAHS. Therefore, the study of the cardiopulmonary function of patients with OSAHS is critical.

Currently, the treatment for moderate and severe OSAHS patients at home and abroad is personalized comprehensive treatment, and the first-line treatment is still transnasal continuous positive pressure ventilation (CPAP) [8]. However, for various reasons, some patients cannot tolerate CPAP. Therefore, for patients unwilling to accept or cannot tolerate CPAP therapy, surgical treatment still plays a positive role in alleviating the degree of upper airway obstruction and improving the patients' clinical symptoms. In addition, most OSAHS patients have multiple plane strictures such as a nasal cavity, palatopharynx, and tongue, which may pose risks during upper airway surgery. Therefore, the choice of surgical methods for such patients must be considered. In this study, 70 patients diagnosed with moderate to severe OSAHS by polysomnography (PSG) and treated with simultaneous multi-plane surgery were retrospectively analyzed, and the effects of simultaneous multiplane surgery on the cardiopulmonary function of middle-aged and young patients with moderate to severe OSAHS were investigated by cardiopulmonary function test.

## 2. Materials and Methods

### 2.1. Research Object

Seventy patients with moderate to severe OSAHS underwent PSG monitoring in our hospital from July 2017 to February 2021 and met the inclusion criteria of this study, including 40 males and 30 females. The following are the inclusion criteria: (1) young and middle-aged patients diagnosed with moderate to severe OSAHS, according to the 2009 guidelines for OSAHS Diagnosis and Surgical Treatment, who underwent PSG examination in our hospital; (2) all patients with preoperative routine physical examination, nasal endoscopic (Ekoda, VET-9001) examination, fiber laryngoscopy (WuScope) and Muller test, upper airway CT(EMERSON) three-dimensional reconstruction and nasal resistance testing, AG200 occlusion plane positioning system (Yicheng Hengda, GSN30087) comprehensive evaluation block plane, at least with nasal planum, velopharyngeal plane, and glossopharyngeal plane two or more stenotic obstruction; (3) no serious maxillofacial malformation, severe coronary heart disease, cerebral apoplexy, malignant tumor, mental disease, severe liver and kidney function, or cardiopulmonary insufficiency; and (4) patients who refused or could not tolerate transnasal continuous positive pressure ventilation and follow-up interruption.

### 2.2. PSG Detection

Sandman Elit (Ty-Co, Canada) and Compumedics ESeries-Polysomnography (Compumedics, Australia) were used to monitor alcohol and tea, caffeine, tranquilizers, or hypnotics during the first 24 h, and the monitoring recording time was >7 h. Electroencephalogram (EEG), ophthalmogram (OGG), maxillofacial emg (EMG), thermosensitive and pressure oral-nasal airflow, snoring, chest and abdominal respiratory movement, electrocardiogram (ECG), blood oxygen saturation, and body position and leg movement before tibial of both lower limbs were collected from all patients. PSG-related indexes, including apnea-hypopnea index (AHI), the lowest blood oxygen saturation (SaO_2_), and percentage of time with oxygen saturation < 90% in total sleep time (TS90%), were analyzed according to the 2007 AASM sleep and respiratory event analysis standard.

### 2.3. Operation Method

Simultaneous multiplane surgery was performed, according to upper airway CT (EMERSON) and routine pharyngeal morphology examination, preoperative personalized evaluation, two or three planes of simultaneous surgical treatment. Details are as follows:

#### 2.3.1. Nasal Plane and Nasal Dilation [9]

(1) Correction of nasal septum deviation. On the premise of preserving nasal septum cartilage autologous as much as possible, the cartilage part at the junction of cartilage and bone was pruned, the bony part of the nasal septum was removed, and the obvious deviated nasal septum cartilage was reduced by scratches on the concave side, or part of the curved cartilage was removed. (2) For the treatment of inferior turbinate hypertrophy, according to the preoperative coronal CT of the sinus, the feasible cryogenic plasma perforation ablation of inferior turbinate mucosal hypertrophy was performed. If the inferior turbinate bone is moved inward, the inferior turbinate fracture can be moved outward to expand the adequate ventilation volume of the nasal cavity. (3) For the abnormal middle turbinate treatment, the vesicular middle turbinate was treated with lateral hemectomy. The inverted deviated middle turbinate was fixed inward.

#### 2.3.2. Oropharyngeal Plane, Striving for Minimally Invasive Treatment, Preserving Normal Mucosa as Far as Possible, and Low-Temperature Plasma-Assisted Palatopharyngoplasty (H-UPPP) Were Selected [10]

Firstly, bilateral tonsil excision was performed by extrapentaminal ablation using the model 8872 low-temperature plasma knife (Arthrocare System, USA), and the anterior and posterior arches were sutured with no. 7 silk thread to close the tonsil fossa. Then, the model 8872 knife head was used to dissect the palatal sail space and ablate the adipose tissue in the space. Then, the model 4855 knife head was used for ablation from both sides of the uvula root to the hard palate, with two holes on each side. Finally, the soft palate and uvula mucosa were sutured in front and back, respectively, and the lengthy uvula was trimmed.

#### 2.3.3. Tongue Plane, Tongue Root, and Tongue Body Ablation [11]

The model 4855 knife head was ablated at 3 points from back to forward in the middle line of the tongue, 5 mm in front of the blind hole, with each point 1 cm apart and 1.5 cm deep into the tongue tissue. The ablation power was 4 W, and the ablation time was 15 s. Two holes were drilled at each side of the tongue. Tonsil hypertrophy of the tongue base was ablated with a model 8872 knife.

### 2.4. Observation Index and Efficacy Evaluation

#### 2.4.1. Static Lung Function Index

Before intervention and 6 months after intervention, the Master Screen pulmonary function detector made by Yeager routinely monitored static lung function indexes of patients: forced expiratory volume in one second/prediction percentage (FEV1 %), forced expiratory volume in one second/forced vital capacity ratio (FEV1/FVC), residual volume (RV), inspiratory capacity (IC), and residual volume/total lung capacity (RV/TCL). Each index was repeated for three times, and the highest value was selected for statistical analysis.

#### 2.4.2. Dynamic Cardiopulmonary Function Index

Static lung function monitoring was followed by resting for 20 min. A cardiopulmonary exercise test (CPET) was performed on a bicycle under electromagnetic braking. Quark PFT Ergo Multifunctional lung test (COSMED) was adopted. Data were recorded every 10 seconds, including the peak maximum oxygen uptake/prediction percentage (Peak VO_2_ %), maximum oxygen uptake/prediction percentage (VO_2_ Max %), peak oxygen pulse/prediction percentage (peak O_2_ Pulse %), oxygen uptake/work rate (VO_2_/WR), ventilatory equivalent for carbon dioxide output (VE/VCO_2_), anaerobic threshold (AT), and maximal ventilation per minute/Maximal Voluntary Ventilation (VEmax/MVV).

#### 2.4.3. Impulse Oscillating Lung Function Technology (IOS) Indicators

The IOS indicators include total respiratory Impedance (Zrs), Rc (Central Resistance), Rp (Peripheral Resistance), 5 Hz respiratory Resistance (Resistance 5, R5), 20 Hz respiratory Resistance (R20), surrounding airway Resistance (R5-R20), 5 Hz (Reactance 5, X5), 20 Hz (Reactance 20, X20), and Resonance Frequency (Resonance Frequency, Fres) to analyze the correlation between the condition of patients with sleep apnea before and after surgery and pulse oscillating lung function indexes.

#### 2.4.4. Echocardiographic Examination Indicators

The echocardiographic examination indicators include Left Ventricular Ejection Fraction (LVEF), Left Ventricular Posterior Wall, LVPW, Left Ventricular Internal Diameter at end-diastole (LVIDd), Interventricular Septum (IVS), Right Ventricular Diameter (RVD), Left Atrial Diameter (LAD), and the calculated Left Ventricular Mass Index (Left Ventricular Mass Index (LVMI)) to analyze the correlation between the condition of sleep apnea patients before and after surgery and cardiac function indicators.

### 2.5. Statistical Analysis

SPSS 17.0 (IBM Corporation, USA) was used for analysis. Quantitative data were expressed by mean ± standard error, and a paired *T*-test was used to analyze and compare the indicators before and after treatment. *P* < 0.05 indicates statistically significant difference.

## 3. Results

From July 2017 to February 2021, 70 patients who received surgical treatment in our department with complete postoperative follow-up data were counted. There were 40 males and 30 females aged from 26 to 59 years. Among the 70 patients, 27 underwent nasal dilatation+low-temperature plasma-assisted velopharyngoplasty+tongue root and tongue plasma-assisted velopharyngoplasty, and 24 underwent nasal dilatation+low-temperature plasma-assisted velopharyngoplasty. Nineteen patients underwent low-temperature plasma-assisted palatopharyngoplasty plus volume reduction of tongue root and tongue.

### 3.1. ESS Scores of Patients before and after Surgery

The results showed that the ESS score decreased significantly 6 months after surgery compared with that before surgery, and the percentage of time when blood oxygen saturation was less than 90% in the total sleep time (TS90 %) also decreased significantly (*P* < 0.01). See Table 1.

### 3.2. Comparison of Static Lung Function Indexes before and after Operation

After surgery, the percentage of forced expiratory volume in the first second (FEV1%) increased from 77.63 ± 1.45% to 84.87 ± 1.20%, and the ratio of forced expiratory volume in the first second to forced lung viability (FEV1/FVC) increased from 66.47 ± 1.90% to 76.04 ± 1.58%, mean increase in deep inspiratory volume (IC) from 2.54 ± 0.16 L to 3.18 ± 0.16 L, and mean percentage of residual (RV/TCL) from 49.71 ± 2.08% to 57.6 ± 1.99%. All of them improved (*P* < 0.01). The mean residual volume (RV) decreased from 98.31 ± 2.39 L to 79.61 ± 1.90 L (*P* < 0.01). The above results indicated that the static cardiopulmonary function of moderate and severe OSAHS patients was improved after multiplane surgery, as shown in Table 2.

### 3.3. Comparison of Dynamic Cardiopulmonary Function Indexes before and after the Operation

After surgery, the percentage of maximal oxygen uptake (VO2 Max %) increased from 78.8 ± 1.38%to 81.14 ± 1.41% (*P* > 0.05). The percentage of peak oxygen uptake to the predicted value (peak VO2%) increased from 80.51 ± 1.57%to 84.39 ± 1.36% on average. The average percentage of peak O2 pulse to predicted value (PEAK O2 Pulse %) increased from 76.33 ± 1.63%to 83.63 ± 1.41%, and the average oxygen power ratio (VO2/WR) increased from 8.06 ± 0.52%to 10.67 ± 0.47%. The mean anaerobic threshold (AT) increased from 48.94 ± 2.17 L/min to 58.34 ± 2.15 L/min, and the mean maximum ventilate/maximum movement ventilate (VEmax/MVV) increased from 75.19 ± 1.45%to 81.73 ± 1.37%. CO_2_ aeration equivalent (VE/ VCO_2_) decreased from 27.07 ± 1.43%to 21.23 ± 1.35% on average (*P* < 0.01), as shown in Table 3. These results indicate that dynamic cardiopulmonary function is improved in patients with moderate to severe OSAHS after multi-plane surgery.

### 3.4. Comparison of AHI and SaO_2_ in Patients before and after the Operation

After surgery, the mean minimum blood oxygen saturation (SaO_2_) increased from 85.33 ± 0.79%to 95.19 ± 0.19% (*P* < 0.01), the mean apnea-hypopnea index (AHI) decreased from 27.44 ± 1.30 times/h to 14.37 ± 0.67 times/h. The AHI and SaO_2_ were improved after operation (*P* < 0.01). See Table 4.

### 3.5. Comparison of IOS Index of Patients before and after Surgery

Among the indicators of pulse oscillating lung function, Rc and R20 mainly reflect the upper airway resistance of patients, among which Rc reflects the viscosity resistance of the large airway, thorax, and diaphragm of the respiratory system. R20 represents the impedance when the oscillation frequency is 20 Hz, mainly reflecting the central respiratory resistance. Zrs mainly reflects the viscosity resistance of the respiratory system, and its main component is airway resistance. R5 represents the impedance at an oscillation frequency of 5 Hz, reflecting the total respiratory resistance, mainly airway resistance. There was no significant difference in Zrs and R5 indexes before and after surgery, but there was a decrease in Zrs and R5 indexes after surgery compared with before surgery. There were statistically significant differences in R20 and Rc before and after surgery (*P* < 0.01), and R20 after surgery was lower than before, as shown in Table 5.

### 3.6. Indexes of Cardiogram before and after Operation

Left posterior ventricular wall, left ventricular end-diastolic diameter, left atrial diameter, and LVMI were indicators reflecting left ventricular structure. The left ventricular end-diastolic diameter and left atrial diameter differed before and after surgery (*P* < 0.01), as shown in Table 6.

## 4. Discussion

Patients with severe OSAHS have recurrent apnea or reduced breathing range during sleep. The basic pathophysiology is repeated intermittent hypoxia during sleep, sleep fragmentation, and frequent microawakenings, resulting in daytime sleepiness, fatigue, inattention, and cognitive decline, thus significantly reducing work efficiency and quality of life [12–16]. Clinical treatment for moderate to severe OSAHS patients is mainly CPAP therapy. Due to severe upper airway stenosis in moderate and severe OSAHS patients, there may be multifaceted obstruction, and the inspiratory pressure of CPAP required for treatment is high, which is difficult for patients to bear and even interferes with sleep, leading to low compliance of CPAP therapy [17, 18]. Therefore, surgical relief of patients with upper airway stenosis or obstruction decreased airway resistance and adverse respiratory events during sleep breathing.

There are few studies on cardiopulmonary function changes in patients with OSAHS. Cardiopulmonary function tests have found that cardiac function changes can occur in patients with severe OSAHS at the reference stage, and both heart and lung functions are changed at the peak stage [19]. Domestic and foreign studies on the changes in lung function in OSAHS patients are still controversial. Zerah-Lancer F's study concluded that MEF50 in the OSAHS group was lower than that in the control group; that is, OSAHS patients presented with pulmonary ventilation dysfunction with reduced midexpiratory airflow velocity [20]. In similar studies, functional residual air capacity, maximum vital capacity, forced vital capacity, expiratory volume at the end of 1 second, and MEF50 were all lower than those in the control group. There were more abnormal lung function indicators than those in Zerah-Lancer F's study [21]. Some scholars have studied the difference in forced lung capacity, forced expiratory volume at the end of 1 second, and MEF25-75 between the OSAHS patients' group and the snoring group with statistical significance [22]. A recent study has highlighted the effect of H-UPPP combined with nasal dilatation in treating OSAHS. They found that the AHI, ESS, and other indicators of patients improved after the operation, and there was no significant increase in the incidence of complications. They believed the combined operation could be a routine treatment for OSAHS [23].

This study's patients with moderate to severe OSAHS underwent multiple planar surgeries simultaneously. Epworth Sleepiness Scale (ESS) scores were compared before and after surgery to observe the surgical efficacy and detect the changes in the cardiopulmonary function of patients before and after surgery. The static and dynamic indexes of cardiopulmonary function, respiratory disturbance index (AHI), and blood oxygen saturation (SaO_2_) were compared before and after the operation. After surgery, all the indexes of static lung function of the patients were improved compared with that before surgery, and the percentage of maximal oxygen uptake peak to the predicted value, percentage of oxygen pulse to the predicted value, the ratio of oxygen uptake power, anaerobic threshold, and maximum ventilatory capacity per minute/maximum exercise volume was increased compared with that before surgery, and AHI and SaO_2_ were improved compared with that before surgery. In addition, this study's results indicate differences in lung function changes in patients with OSAHS before and after surgery, and the changes in lung function are reflected in the increase of airway resistance, in which the increase in upper airway resistance is more prominent. In this study, the indexes of left ventricular end-diastolic diameter and left atrial diameter were higher before and after surgery. These results showed that the changes in cardiac structure in patients with OSAHS were mainly manifested as the changes in left cardiac structure, and the changes in cardiac function were mainly manifested as the decline of left diastolic function, which was consistent with domestic and foreign reports [24–26]. This study suggests that it is feasible for patients with OSAHS who are unable to tolerate or unwilling to undergo noninvasive assisted ventilation therapy to undergo simultaneous multiplane stenosis surgery. It could reduce clinical symptoms and improve cardiopulmonary function. The follow-up time of this study is not long enough, and the number of cases is small, so long-term observation with large sample size is needed for long-term efficacy.

## Figures and Tables

**Table 1:** Comparison of ESS and TS90% before and after the operation.

Observation indicator	Group		
	Before operation	After operation	*P* value
ESS (score)	11.90 ± 0.62	9.50 ± 0.51	<0.001
TS90 % (%)	0.49 ± 0.04	0.33 ± 0.03	<0.001

**Table 2:** Comparison of static lung function indexes before and after surgery.

Observation indicator	Group		
	Before operation	After operation	*P* value
FEV1 % (%)	77.63 ± 1.45	84.87 ± 1.20	<0.01
FEV1/FVC (%)	66.47 ± 1.90	76.04 ± 1.58	<0.01
IC (L)	2.54 ± 0.16	3.18 ± 0.16	<0.01
RV (L)	98.31 ± 2.39	79.61 ± 1.90	<0.01
RV/TLC (%)	49.71 ± 2.08	57.6 ± 1.99	<0.01

**Table 3:** Comparison of dynamic pulmonary function indexes before and after surgery.

Observation indicator	Group		
	Before operation	After operation	*P* value
Peak VO_2_ % (%)	80.51 ± 1.57	84.39 ± 1.36	<0.01
Peak O_2_ plus % (%)	76.33 ± 1.63	83.63 ± 1.41	<0.01
VO_2_/WR (%)	8.06 ± 0.52	10.67 ± 0.47	<0.01
AT (L/min)	48.94 ± 2.17	58.34 ± 2.15	<0.01
VE/VCO_2_ % (%)	27.07 ± 1.43	21.23 ± 1.35	<0.01
VEmax/MVV (%)	75.19 ± 1.45	81.73 ± 1.37	<0.01

**Table 4:** Comparison of AHI and SaO_2_ in patients before and after the operation.

Observation indicator	Group		
	Before operation	After operation	*P* value
SaO_2_ (%)	85.33 ± 0.79	95.19 ± 0.19	<0.01
AHI (times/h)	27.44 ± 1.30	14.37 ± 0.67	<0.01

**Table 5:** Comparison of IOS indexes before and after surgery (KPa∗L-1∗ SEC-1).

Observation indicator	Group		
	Before operation	After operation	*P* value
Zrs	0.50 ± 0.03	0.48 ± 0.03	0.12
Rc	0.26 ± 0.02	0.22 ± 0.02	<0.01
R5	0.47 ± 0.04	0.45 ± 0.03	0.15
R20	0.34 ± 0.02	0.29 ± 0.02	<0.01

**Table 6:** Comparison of IOS indicators before and after surgery.

Observation indicator	Group		
	Before operation	After operation	*P* value
Left ventricular end-diastolic diameter (mm)	51.41 ± 1.62	44.51 ± 1.49	<0.01
Left atrial diameter (mm)	42.63 ± 1.71	39.40 ± 1.75	<0.01
Left ventricular posterior wall (mm)	9.11 ± 0.39	9.08 ± 0.38	0.85
LVMI (g∗m^−2^)	78.52 ± 1.29	78.03 ± 1.36	0.12

## Data Availability

The data used to support the findings of this study are available from the corresponding author upon request.
